# Changes in threats from chronic obstructive pulmonary disorder and lung cancer with environmental improvements in China: Quantitative evaluation and prediction based on a model with age as a probe

**DOI:** 10.1016/j.heliyon.2024.e28977

**Published:** 2024-04-02

**Authors:** Liu Hui

**Affiliations:** College of Medical Laboratory, Dalian Medical University, Dalian, 116044, China

**Keywords:** Environmental risk, Chronic disease, Noncommunicable diseases, Mortality, Disease management, Risk assessment

## Abstract

Various indicators can be used to assess threats from chronic diseases. This study presented new indicators of quantitative evaluation and prediction of threats from chronic obstructive pulmonary disorder (COPD) and lung cancer and assessed relevant changes in these indicators occurring with environmental improvements. Age at zero mortality (AM0) and age at average mortality (AMa) values were calculated based on the regression of the linear relationship of age with mortality for COPD or lung cancer. The lower the AM0 or AMa of a chronic disease, the greater the threats from the disease to a population were considered to be. AM0 values of both diseases were higher in 2019 than in 2004. Moreover, AM0 was lower for lung cancer than for COPD (0.365 vs. 41.643); however, lung cancer and COPD demonstrated almost identical values for age-standardized mortality. AMa values of both the diseases in 2004 and 2019 were within the range of the median age group (70–74 years). In recent years, the overall mortality risk for lung cancer and COPD has decreased with environmental improvement, and aging has played a major role in lung cancer and COPD development. AM0 and AMa values may be used as a theoretical basis for further research on chronic diseases, particularly lung cancer and COPD.

## 1 Introduction

Chronic obstructive pulmonary disease (COPD) and lung cancer are prevalent chronic respiratory diseases, and environmental factors strongly impact their occurrence, development, and outcome. Although they demonstrated some similarities, COPD and lung cancer have several distinct characteristics, in terms of both their etiology and progression. As such, understanding their common and distinct risk factors is crucial for effective prevention, diagnosis, and treatment of COPD and lung cancer. Prolonged exposure to environmental pollutants, such as smoke, air pollution, and occupational hazards (e.g., asbestos), can increase COPD and lung cancer risks [[1], [2], [3]]. The primary cause of lung disease due to environmental pollution is inhalation of airborne harmful particles and gases. One of the most common pollutants leading to lung disease is particulate matter, which when inhaled, can penetrate deep into the lungs and cause inflammation. It can lead to respiratory problems such as asthma, chronic bronchitis, or even lung cancer. Other pollutants involved in lung disease development include nitrogen dioxide, sulfur dioxide, ozone, and carbon monoxide. These pollutants can also cause airway irritation and inflammation, resulting in inflammation and damage over time.

Aging, a natural, inevitable process, affects every aspect of the human body, including the lungs. With aging, the lungs undergo structural changes, which can impair their function. These changes include decreases in lung tissue elasticity—impeding efficient lung expansion and contraction, reducing lung capacity, and hampering effective lung oxygen–carbon dioxide exchange. Aging also affects the immune system by gradually weakening it. Therefore, compared with younger individuals, older individuals are more susceptible to respiratory infections, such as pneumonia, which can further contribute to lung disease development.

Improvements in socioeconomic and environmental conditions have increased the longevity of older populations globally. However, the development of chronic diseases, including respiratory chronic diseases, is generally driven by aging and nonaging factors [[4], [5], [6]]. Aging is an omnipresent temporal variable for all living organisms, affecting the basal levels of health. Nonaging factors are related to genetics, the environment, and medical treatments. They are temporal, with their importance and strength changing with time. Aging and many nonaging factors can increase mortality related to some chronic diseases—inconsistent with the increasing life expectancy in developed societies [7,8]. Thus, assessing the degrees of threat from and burden of different chronic diseases, such as COPD and lung cancer, present to health and survival is warranted.

Diseases are considered detrimental if they primarily shorten survival in younger individuals. These diseases may predominantly be caused by nonaging factors; moreover, compared with diseases caused by aging factors, these diseases may have more control strategies available. Therefore, a comprehensive analysis of the threats from these diseases to individuals of different ages can facilitate the development of not only efficient public health strategies but also targeted treatment programs; it can also aid in selecting appropriate palliative care strategies.

The standardized proportion of dying of a specific cause—not affected by the population composition—is commonly used to evaluate the disease's risk in an affected population [7,8]. However, for the assessment of survival threats from a chronic disease, factors related to not only a relatively young population but also the total population should be considered. The lower the age at death, the greater are the effects of nonaging factors and risks to the population; as such, age may be considered a sensitive marker of threats from chronic diseases.

In this study, by using 2004 and 2019 data from China's National Disease Mortality Surveillance System, the occurrence of COPD and lung cancer was analyzed quantitatively, with age as a probe. In particular, through a comparison of 2004 and 2019 data related to different diseases and social development levels, the patterns of the occurrence of COPD and lung cancer were established. These patterns were used to predict threats from COPD and lung cancer and assess the effectiveness of the relevant current prevention and treatment measures.

## 2 Materials and methods

### 2.1 Raw data extraction

Raw data regarding lung cancer and COPD for 2004 and 2019 were obtained from the National Disease Mortality Surveillance System of the Chinese Center for Disease Control and Prevention (Table 1, Table 2) [9,10]. These data included information from more than 73 million Chinese individuals. To determine mortality statistics. International Classification of Diseases 10th Revision codes [11] for lung cancer (C33–C34) and COPD (J40–J44) were used.

**Table 1:** Age-stratified mortality rates for lung cancer and COPD in monitored Chinese population in 2004 and 2019 (annual deaths per 10^5^ population).

Age group	2004		2019		Population	
	Lung cancer	COPD	Lung cancer	COPD	2004	2019
55∼	65.93	65.56	58.44	12.85	2957812	17445735
60∼	101.48	140.06	98.20	32.08	2486122	17480461
65∼	158.21	302.40	164.00	76.53	2125649	14072230
70∼	247.31	667.63	244.28	189.85	1601637	8860096
75∼	297.73	1216.94	340.44	427.35	1022733	5795999
80∼	321.61	2248.32	382.68	818.06	545697	4124288
>85∼	301.53	3405.99	528.22	2287.25	308427	2146285
Average mortality	158.64	522.83	170.09	204.56	–	–
Standardized mortality^a^	27.41	76.21	26.86	26.44	–	–

a Includes mortality in all age groups from 0 to 5 years to >85 years standardized using 2000 data.

**Table 2:** Age- and sex-stratified mortality rates for lung cancer and COPD in monitored Chinese population in 2019 (annual deaths per 10^5^ population).

Age group	Lung cancer		COPD		Population	
	Men	Women	Men	Women	Men	Women
55∼	86.42	30.21	19.04	6.60	8760381	8685354
60∼	146.61	49.25	46.06	17.40	8789447	8691014
65∼	249.05	82.52	109.60	44.86	6884845	7187385
70∼^a^	367.53	127.47	260.29	123.10	4310883	4549213
75∼	498.85	197.69	582.10	287.89	2747293	3048706
80∼	554.92	247.48	1093.40	601.90	1813789	2310499
>85∼	752.20	375.93	2773.04	1956.98	868651	1277634
Average mortality	245.06	98.41	246.95	163.91	–	–

a Median age group.

### 2.2 Model of COPD and lung cancer mortality with age as the probe

For the current model, the basic assumptions for the model were used:

(1) The relationship between age (i.e., different age groups) and mortality is linear because of the roles of risk factors for death, including aging.
(2) Aging plays a key role in deaths in individuals aged >60 years.

A regression equation was used to confirm the linear relationship between median age in different age groups on the *y* axis and natural logarithm of mortality [ln(mortality)] from COPD or lung cancer on the *x* axis. The coefficient of determination (*R*^2^) of linear regression was determined, which indicated the roles of risk factors for death. An *R*^2^ of <0.9 was considered to suggest that a random risk factor rather than cumulative risk factor, such as an accident, plays a crucial role in lung cancer or COPD development.

The linear regression used SPSS software (SPSS, Chicago, IL, USA). A value of P < 0.01, was considered as statistically significant.

### 2.3 Calculation of age mortality

Next, this study developed a new index for comprehensive analysis of threats from diseases to individuals of different ages.

Age at zero mortality (AM0) for a disease is defined as the age at which 10^−5^ deaths occur from the disease over 1 year; moreover, age at average mortality (AMa) for a disease is defined as the age at which average mortality occurs from the disease among the observed age groups over 1 year. The intercept of the linear regression in the current model was considered to indicate AM0. AM0 represents greater weight to threats from a disease in younger age groups. The lower the AM0 of a disease, the greater is the threat it poses to the affected population.

AMa was calculated using the regression equation between age and mortality (i.e., AMa = *f*(*x*); *x* was average mortality in Table 1). In theory, AMa, indicating that aging plays a major role in deaths, should be within the range of the median age group; it was 70–74 years in the present study. Therefore, AMa <70 was considered to indicate that threats from a disease are mainly due to nonaging factors, whereas AMa >74 was considered to denote that protective factors are mainly due to delaying aging.

## 3 Results

This study created graphs demonstrating the linear relationship of ln(mortality) with median age (*r*^2^ = 0.998; *p* < 0.001); Fig. 1 illustrates an example graph created using data of total COPD population in 2019.

**Fig. 1:** Linear relationship between COPD mortality and age in 2019.

AM0, AMa, and *R*^2^ values for COPD and lung cancer in 2004 and 2019 are listed in Table 3; moreover, sex-stratified AM0, AMa, and *R*^2^ values for COPD and lung cancer in 2019 are presented in Table 4. AM0 was considered to indicate average threats in our populations. For both diseases, AM0 was greater in 2019 than in 2004, suggesting that threats from either of the two diseases were lower in 2019 than in 2004. Similarly, regardless of the year, AM0 was greater in women than in men, suggesting that threats from either of the two diseases were lower in women than in men.

**Table 3:** *R*^2^, AM0, and AMa values in 2004 and 2019.

Disease	R^2^		AM0		AMa	
	2004	2019	2004	2019	2004	2019
Lung cancer	0.872	0.966	−12.987	0.365	69.453	69.418
COPD	0.991	0.998	25.271	41.643	71.496	72.962

AM0, age at zero mortality; AMa, age at average mortality; *R*^2^, coefficient of determination.

**Table 4:** Sex-stratified *R*^2^, AM0, and AMa values in 2019.

Disease	R^2^		AM0		AMa	
	Men	Women	Men	Women	Men	Women
Lung cancer	0.957	0.990	−5.823	15.494	69.053	70.018
COPD	0.998	0.998	38.655	46.686	72.206	74.064

AM0, age at zero mortality; AMa, age at average mortality; *R*^2^, coefficient of determination.

In both 2004 and 2019, AMa for both diseases was almost within the range of the median age group (70–74 years), indicating that aging has a major role in deaths due to either of the diseases. Notably, *R*^2^ was <0.9 for lung cancer in 2004, suggesting that random risk factors played crucial roles in lung cancer occurrence in 2004.

## 4 Discussion

Over 2015–2019, China's clean air policies have led to improvements in air quality [[12], [13], [14]], along with significant reductions in ambient levels of particulate matter with a diameter of <1, <2.5, and <10 μm [12]. Moreover, volatile organic compound emission decreased from its peak at 16.40 Tg in 2016 to 15.72 Tg in 2019 [15]. COPD and lung cancer are major chronic respiratory diseases, and their occurrence is affected by environmental factors [[1], [2], [3]]. Therefore, the current study included 2004 and 2019 data for the two aforementioned diseases from China's National Disease Mortality Surveillance System.

When discussing threats from a chronic disease to survival, factors related to both the total population and a relatively young population should be considered. Therefore, here, AM0 and AMa were used for comprehensive analyses of threats from COPD and lung cancer among individuals of different ages. COPD and lung cancer are typical diseases caused by environmental and aging-related factors. When environmental factors are the main risk factors for a chronic disease, the mortality rate in younger individuals tends to be high, with a low AM0; threats from this disease may be high, and the strategy to control this disease may be based on environmental improvements. When aging is the main risk factor for a chronic disease, AM0 is high with an older overall average age at death; threats from this disease to the total population may be low, with most deaths occurring due to natural causes. Moreover, the strategy to control this disease may be based on improving the general health status and delaying aging or aging-related death. This is the first study thus far assessing threats from the chronic diseases COPD and lung cancer in different age groups, based on AM0 and AMa.

Regression analysis of the linear relationship between AM0 or AMa and mortality was conducted to estimate the age of mortality from COPD or lung cancer. Here, AM0 or AMa was not affected by the different age compositions of the population; therefore, the calculated values were representative of any of the considered populations. The threats based on AM0 appeared to be more accurate than those based on age-standardized mortality rates: When the age-standardized mortality rate was used as the indicator, threats from lung cancer in 2019 and 2004 were similar (27.41 and 26.86, respectively); however, when AM0 was used as the indicator, threats from lung cancer were significantly lower in 2019 than in 2004 (−12.987 vs. 0.365). In general, AM0 was noted to allow for an accurate judgment of threats from a disease specifically in younger age groups.

In the present study, AM0 was greater in women than in men for both COPD and lung cancer, suggesting that threats from the two diseases were greater in men than in women [[16], [17], [18]] and that AM0 is a reasonable predictor for mortality. This was possibly due to a considerable proportion of men smoking cigarettes.

For both chronic disorders, threats evaluated using AM0 demonstrated changes with environmental improvements. Furthermore, in 2019, age-standardized mortality was similar for COPD and lung cancer (26.86 and 26.44, respectively), whereas AM0 was higher for lung cancer than for COPD (0.365 vs 41.643); this was possibly because of threats from lung cancer being greater in younger individuals.

Notably, the *R*^2^ for lung cancer was <0.9 in 2004 and > 0.9 in 2019. Thus, random risk factors may have played a major role in lung cancer development in 2004, and these risk factors may underlie the positive changes related to environmental improvements. For both COPD and lung cancer, AMa in both 2004 and 2019 were almost within the range of the median age group (70–74 years). Therefore, aging plays a major role in mortality related to COPD and lung cancer. However, the AMa of lung cancer was approximately 70. In general, the AMa-based assessment of overall threats from lung cancer indicated that nonaging factors have a considerable role in lung cancer development. Moreover, although more men than women smoke cigarettes in China [[16], [17], [18]], the differences in AMa values between men and women were not large. Thus, environmental improvement may have a critical role in reducing threats from COPD and lung cancer.

A limitation of this study is that other variables, such as height, weight, body mass index, and occupational history, were not controlled for. These factors tend to change as society progresses and should be included in quantitative analyses of particular issues.

In summary, this study used AM0 and AMa to analyze threats from COPD and lung cancer among Chinese individuals in 2004 and 2019. AM0 is suitable for evaluating threats from a disease, whereas AMa aids in assessing the roles of aging and nonaging-related risk factors for the disease. AM0 and AMa can be used to efficiently detect whether the disease is mainly caused by aging factors. When present as a main risk factor, aging indicates that threats from a disease are related to death by natural causes. Moreover, for this disease, the control strategy should involve improving the general health status and delaying aging or aging-related death. In other words, AM0 and AMa can explain different aspects of mortality in a disease. In recent years, environmental improvement has reduced the overall threats from lung cancer and COPD, and aging has played an important role in lung cancer and COPD development. As such, understanding the aforementioned threat indicators may provide a theoretical basis for further research on chronic diseases, such as lung cancer and COPD, and the relevant effects of environmental improvement.

## CRediT authorship contribution statement

**Liu Hui:** Writing – review & editing, Writing – original draft, Formal analysis, Data curation, Conceptualization.

## Declaration of competing interest

The authors declare that they have no known competing financial interests or personal relationships that could have appeared to influence the work reported in this paper.
